The article "Effects of Mind Mapping Combined with Microvideo Explanation on Disease Perception Control and Nursing Cooperation during Membrane Induction Therapy in Patients with Infectious Nonunion after Tibial Trauma" was retracted in 2024. Reasons: signs of a paper mill; suspected computer-generated content; unreliable results or conclusions; lack of ethics approval or compliance.

# Effects of Mind Mapping Combined with Microvideo Explanation on Disease Perception Control and Nursing Cooperation during Membrane Induction Therapy in Patients with Infectious Nonunion after Tibial Trauma

**DOI:** 10.1155/2022/4439595

**Published:** 2022-06-17

**Authors:** Rui Xiong, Ni Wang, JingXuan He

**Affiliations:** Department of Orthopedics, General Hospital of the Yangtze River Shipping, Wuhan, Hubei 430010, China

## Abstract

**Objective:**

To study the effects of mind mapping combined with microvideo explanation on disease perception control and nursing cooperation during membrane induction therapy in patients with infectious nonunion after tibial trauma.

**Methods:**

30 patients with infectious nonunion after tibial trauma treated in the hospital between March 2018 and March 2022 were selected as the research subjects, and the patients were divided into a control group (*n* = 15) and an observation group (*n* = 15) by the random number table method. During membrane induction therapy, the control group adopted a routine nursing method while the observation group was given a nursing method of mind mapping combined with microvideo explanation. The disease perception control, nursing cooperation, and self-care ability of the two groups of patients were compared.

**Results:**

After nursing, the scores of aspects of “life impact (3.87 ± 0.92),” “duration (3.20 ± 1.01),” and “emotions (3.93 ± 0.59)” of the Brief Illness Perception Questionnaire (B-IPQ) in the observation group were lower than those in the control group (5.27 ± 0.88, 4.67 ± 1.05, and 4.93 ± 0.80, respectively) (*P* < 0.05) while the scores of “self-control (6.80 ± 1.21)” and “disease awareness (7.27 ± 0.70)” were higher than those in the control group (5.00 ± 1.07 and 5.93 ± 0.70, respectively) (*P* < 0.05). There was no significant difference in the total compliance rate between the two groups (*P* > 0.05). After nursing, the scores of dimensions and the total score of the Exercise of Self-Care Agency Scale (ESCA) were increased in the two groups, and the scores were higher in the observation group than those in the control group (*P* < 0.05).

**Conclusion:**

Mind mapping combined with microvideo explanation can improve the disease perception control during membrane induction therapy in patients with infectious nonunion after tibial trauma, improve the self-care ability, and facilitate the smooth progress of treatment.

## 1. Introduction

Infectious nonunion and bone defect are serious complications of trauma orthopedics, which are common after tibial fracture. Patients are often accompanied by local pain, joint dysfunction, deformity, and other uncomfortable symptoms, which seriously affect the daily life of patients [1, 2]. Membrane induction therapy is currently a commonly used surgical method for the treatment of infectious nonunion in clinical practice. This surgical method requires local infection control first, and then reconstruction of the bone defect [3]; the surgical methods are complex and the treatment cycle is long, and the pathogenesis and treatment process of the disease are complex. Patients often fear because of their lack of understanding of the disease, which in turn affects medical compliance behavior and disease prognosis [4]. Previous studies have pointed out that active, scientific, and effective health education methods can improve patients' cognition of diseases, improve patients' disease perception and treatment compliance, and are conducive to disease recovery [5]. However, conventional nursing and health education methods are abstract and difficult to understand. Patients lack understanding of professional vocabulary, and there are still problems of poor communication and inadequate propaganda and education, therefore, the implementation effect needs to be improved. Mind mapping is a technique to visualize abstract things and knowledge, making medical content more straightforward, vivid, and concise, with a clear structure and prominent focus, which is convenient for medical staff, patients, and family members to learn and master [6]. In addition, in recent years, with the development of mobile Internet technology and new media, there are various forms of health knowledge dissemination by means of WeChat, Weibo, and other social platforms using microvideos, short videos, etc. [7, 8]. Compared with the traditional text and picture description, this method is more intuitive and less limited by the cultural level of viewers. As a new educational model, microvideo health education has been applied in clinical nursing work. Therefore, this study explored the effects of mind mapping combined with microvideo explanation on disease perception control and nursing cooperation during membrane induction therapy in patients with infectious nonunion after tibial trauma, aiming to provide a simpler and easier method for clinical trauma orthopaedic education, to improve patient awareness, and the results were now reported as follows.

The article "Effects of Mind Mapping Combined with Microvideo Explanation on Disease Perception Control and Nursing Cooperation during Membrane Induction Therapy in Patients with Infectious Nonunion after Tibial Trauma" was retracted in 2024. Reasons: signs of a paper mill; suspected computer-generated content; unreliable results or conclusions; lack of ethics approval or compliance.

## 2. Materials and Methods

### 2.1. General Information

A total of 30 patients with infectious nonunion after tibial trauma who were treated in our hospital from March 2018 to March 2022 were selected as the research subjects, and the patients were divided into a control group (*n* = 15) and an observation group (*n* = 15) by the random number table method. Among them, there were 10 males and 5 females in the control group; the age ranged from 41 to 54 years, with an average of 46.53 ± 4.22 years; in terms of their educational background, 2 cases have educational background of primary schools, 6 cases have been educated in junior high schools, and 7 cases have been educated in high schools and above. The observation group included 9 males and 6 females, aged 43–58 years, with an average age of 48.80 ± 4.39 years; their educational background covered 3 cases who have been educated in primary schools, 6 cases in junior high schools, and 6 cases in high schools and above. There was no significant difference in the comparison of general data between the two groups (*P* > 0.05), and the groups were comparable.

Inclusion criteria were as follows: (1) all patients who met the diagnostic criteria for infectious nonunion after tibial trauma [9] and were undergoing membrane induction therapy; (2) all who had unilateral limb damage; (3) patients aged ≥18 years; and (4) all patients who have been educated in primary schools or above and were able to understand the scales and questionnaires involved in this research. Exclusion criteria were as follows: (1) patients with mental, communication, comprehension, and hearing impairments; (2) patients who had refused more than 2 times of nursing operations; and (3) patients with major diseases such as malignant tumors and liver and kidney failure.

### 2.2. Methods

Control group: conventional nursing methods were adopted, and the main purpose was to enable patients to master disease knowledge, functional exercise methods to relieve pain, and relieve fear and anxiety: (1) General nursing: ① preoperative guidance: explained membrane induction therapy to patients before surgery; (2) postoperative care: (A) raised the affected limb after operation, promoted venous return, and reduced limb swelling; (B) evaluated patient's pain and diverted patients' attention by chatting with the patients or asking them to listen to music. Patients with severe pain should use analgesics as prescribed by the doctor; (C) observed the bleeding, swelling, and blood circulation of the affected limb at the wound site every day and changed the gauze in time when there was a lot of bleeding and exudate at the wound site. (2) Health education: ① Functional exercise: (A) massaged the limbs every day to promote blood circulation and stability recovery, prevented the formation of deep vein thrombosis in the lower extremities, and reduced edema; (B) ankle joint movement: straightened the ankle joint distally for 3-4 s, then dorsiflexed it distally for 3-4 s, straightened and dorsiflexed it once, and repeated the training about 100 times a day; (C) quadriceps contraction training: kept the lower limbs still and contracted the quadriceps for about 10 s or relaxed after feeling tired. Repeated this 10–20 times each time, and trained 3 to 4 times a day, paid attention to the gradual progress of the training process, as long as patients could tolerate it. ②Dietary care: instructed patients to eat a high-protein, high-nutrition, and high-vitamin diet to supplement their daily energy needs, eat more fresh fruits and vegetables, avoid spicy and greasy foods, and drink more water to prevent the risk of blood clots from increasing blood viscosity. ③ Psychological care: patients often have anxiety and fear because they were worried about the prognosis of the disease and functional recovery. Before the operation, patients should be introduced to the environment, members of the surgical team, related disease knowledge, and previous successful cases, so as to comfort the patients, relieve their tension, encourage them to enhance their confidence in treatment; guided their family members to participate in patients' functional rehabilitation after surgery, encouraged and accompanied patients to improve patients' compliance, and enabled them to actively participate in the treatment process.

The article "Effects of Mind Mapping Combined with Microvideo Explanation on Disease Perception Control and Nursing Cooperation during Membrane Induction Therapy in Patients with Infectious Nonunion after Tibial Trauma" was retracted in 2024. Reasons: signs of a paper mill; suspected computer-generated content; unreliable results or conclusions; lack of ethics approval or compliance.

Observation group: the nursing method using mind mapping combined with microvideo explanation: (1) Established a nursing team: members included 1 chief physician, 1 head nurse, several nurses, 1 rehabilitation therapist, and 1 video technician, and all personnel entered the research group after passing the training. (2) Preparation of mind maps: nurses assessed patients' awareness of the disease and their rehabilitation needs, combined with current nursing deficiencies, on the basis of collecting and reviewing relevant literature, consulted relevant experts, the head nurse and chief physician jointly conducted compilation of mind maps, listened to the relevant suggestions of front-line staff, used relevant software to formulate reasonable and appropriate mind maps, and distributed them to staff and patients so that they could master and learn, as shown in Figure 1. (3) Microvideo production: on the basis of understanding the psychological and physiological needs of patients, nurses consulted literature, collected data, and combined past work experience to conduct targeted video shooting and video production around the possible nursing problems of patients during the perioperative period. Video production was completed under the guidance of video technicians; the content included disease knowledge introduction, preoperative guidance, surgical precautions and key points, postoperative functional exercise methods, and discharge guidance (postoperative rehabilitation functional exercise methods were provided by rehabilitation therapists; they were based on the actual situation of the department and patients with infectious nonunion after tibial trauma nonunion of membrane induction therapy to select the methods for functional exercise); the total duration of each video should not exceed 5 minutes, to ensure that it should be easy to understand, interesting, and scientific; During the treatment of patients, provide guidance through the WeChat group or organize patients to watch, gradually learn perioperative knowledge, and set up medical staff in the group to answer patients' questions for 24 hours.

The article "Effects of Mind Mapping Combined with Microvideo Explanation on Disease Perception Control and Nursing Cooperation during Membrane Induction Therapy in Patients with Infectious Nonunion after Tibial Trauma" was retracted in 2024. Reasons: signs of a paper mill; suspected computer-generated content; unreliable results or conclusions; lack of ethics approval or compliance.

### 2.3. Observation Indicators

(1) Illness perception control: assessed before and after nursing care by using The Brief Illness Perception Questionnaire (B-IPQ) [10], which was developed by Broadbent and included life impact, duration, self-control, treatment control, symptom, attention, disease understanding, emotion, and other items; the first 8 items were scored by a 0–10 scale, items 3, 4, and 7 were scored in reverse, and item 9 is an open-ended question (patients listed three important causes of the disease, which was not mandatory for patients), with a total score of 0 to 80; the higher the score was, the more negative perception the patient has towards the disease. (2) Nursing cooperation: a questionnaire designed by the hospital was used to evaluate patients' compliance, which was divided into three levels: compliance, basic compliance, and noncompliance. The total compliance rate was the sum of the compliance rate and the basic compliance rate. (3) Self-care ability: before and after nursing intervention, the Exercise of Self-Care Agency Scale (ESCA) [11] was used for evaluation, which included self-concept (9 items), self-responsibility (8 items), self-care skill (12 items), and health knowledge level (14 items); in these 4 dimensions with a total of 43 items, each item adopted the Likert 5-level scoring method, ranging from “very similar to me” to “not at all similar to me” with a score of 0∼4, the total score is 172 points, and the higher the score, the stronger the patients' self-care ability.

### 2.4. Data Analysis

SPSS 21.0 software was used for statistical analysis. The count data (%) of normal distribution were tested by the *χ*2 test, and the measurement data ($\bar{x}$ ± *s*) were analyzed by the *t* test. *P* < 0.05 was considered to be statistically significant.

## 3. Results

### 3.1. Comparison of Disease Perception Control

Before nursing, there was no significant difference in the scores of B-IPQ items between the two groups (*P* > 0.05); after nursing, the scores of “life impact,” “duration,” and “emotions” in the observation group were lower than those in the control group (*P* < 0.05), and the scores of “self-control” and “disease awareness” were higher than those of the control group (*P* < 0.05), as shown in Table 1.

The article "Effects of Mind Mapping Combined with Microvideo Explanation on Disease Perception Control and Nursing Cooperation during Membrane Induction Therapy in Patients with Infectious Nonunion after Tibial Trauma" was retracted in 2024. Reasons: signs of a paper mill; suspected computer-generated content; unreliable results or conclusions; lack of ethics approval or compliance.

### 3.2. Comparison of Nursing Cooperation

The compliance rate of the observation group was 100.00%, and the compliance rate of the control group was 93.33%. There was no significant difference in the total compliance rate between the two groups (*P* > 0.05), as shown in Table 2.

### 3.3. Comparison of Self-Care Ability

Before nursing, there was no significant difference in scores of the ESCA dimension between the two groups (*P* > 0.05); after nursing, scores of the ESCA dimension and total scores in the two groups were increased, and scores of the observation group were higher than those of the control group (*P* < 0.05), as shown in Table 3.

## 4. Discussion

At present, the main surgical method for patients with infectious nonunion after tibial trauma is membrane induction therapy, which follows the principle of staged treatment, that is, the infection is controlled first and then the nonunion of the bone defect is treated, so the treatment cycle is long. When the wound is infected, the clinical symptoms of the patients are more serious, which can easily lead to fear and anxiety of patients [12]. Therefore, it is necessary to pay attention to the psychological needs of patients to improve their compliance with treatment and improve the prognosis. Mind mapping used to be one of the tools to improve learning efficiency, and it has the advantages of being intuitive and simple; microvideos are a means of displaying health education knowledge through a video, which is convenient for patients to understand and remember. Mind mapping and microvideos used in nursing teaching, clinical nursing management, health education, and other fields have achieved certain results, which are conducive to the development of clinical nursing [7, 13].

Results of this study showed that after nursing, scores of the observation group were lower than the scores of the control group in terms of “life impact,” “duration,” and “emotion” (*P* < 0.05), and scores of the observation group were higher than scores of the control group in terms of “self-control” and “disease awareness” (*P* < 0.05), which indicated that the use of mind mapping combined with microvideo explanations could improve disease perception control during membrane induction therapy in patients with infectious nonunion after tibial trauma, and improve their awareness of the disease. Nonunion is a serious complication after tibial trauma. Patients' wounds remain unhealed for a long time, and the prolonged course of the disease will affect patients' confidence in recovery. In addition to the inability to heal the wound, patients with infected nonunion may also experience symptoms such as fever, pain in the affected limb, and bone defect, which increases the burden on the patient. Patients often have negative psychology due to fear of the prognosis of the disease (such as amputation, and disability), which may lead to a sense of powerlessness, unable to control the progress of the disease, and then reduce compliance and willingness to cooperate. Mind mapping in this study can simplify, concretize, and make complex pathological knowledge three-dimensional, so that patients and their families can better understand the treatment plan and improve their cognition of the disease to achieve the purpose of disease perception control and help patients overcome their previous ignorance and fear of the disease, and change their distrust of medical staff [14]. At the same time, combined with microvideo explanations, patients can learn about the causes of infectious nonunion, rehabilitation programs, functional exercise methods, dietary guidance, etc. Because microvideos are more intuitive than pictures and text, they are more conducive to patients' learning and memory. Therefore, the scores of “life impact,” “self-control,” and “disease awareness” in the observation group were better than those in the control group. Since the conventional treatment used in the control group also had a certain clinical effect on the patients, the patients' compliance with the nursing intervention did not change much.

The article "Effects of Mind Mapping Combined with Microvideo Explanation on Disease Perception Control and Nursing Cooperation during Membrane Induction Therapy in Patients with Infectious Nonunion after Tibial Trauma" was retracted in 2024. Reasons: signs of a paper mill; suspected computer-generated content; unreliable results or conclusions; lack of ethics approval or compliance.

This study also found that after nursing, scores of the ESCA dimension and total scores in the observation group were higher than those in the control group (*P* < 0.05), which indicated that mind mapping combined with microvideo could improve patients' self-care ability and benefit disease recovery. Mind mapping incorporates pathological knowledge involved in patients' perioperative period, improves patients' cognitive level with targeted nursing methods, guides patients to strengthen self-management, and keeps patients vigilant in medication, diet, rehabilitation exercise, psychological adjustment, etc., thereby improving self-care ability [15]. However, the control group lacked specific and visual guidance, and self-control in medication, rehabilitation, functional exercise, etc. would be slightly weaker; hence, the ESCA score of the patients in the observation group was not as good as that of the patients in the observation group. In addition, the content of health education for infectious nonunion is numerous and complicated. Patients are in pain and have limited activities. They cannot master correct self-care methods in a short time. Microvideos convey complex functional exercises, rehabilitation physiotherapy in an intuitive form, and patients can deepen their impression through repeated viewing. Even after discharge, patients and their families can still conduct self-health education and guidance through microvideos [16], so the patients' self-care ability is higher.

The article "Effects of Mind Mapping Combined with Microvideo Explanation on Disease Perception Control and Nursing Cooperation during Membrane Induction Therapy in Patients with Infectious Nonunion after Tibial Trauma" was retracted in 2024. Reasons: signs of a paper mill; suspected computer-generated content; unreliable results or conclusions; lack of ethics approval or compliance.

In conclusion, mind mapping combined with microvideos can improve disease perception control of patients with infectious nonunion after tibial trauma during membrane induction therapy and improve patients' nursing cooperation and self-care ability, which is conducive to disease recovery.

## Figures and Tables

**Figure 1:** Schematic diagram of mind mapping of infectious nonunion after tibial trauma

**Table 1:** Comparison of B-IPQ scores between the two groups of patients ($\bar{x}$ ± *s*, points).

Group	*n*	Life impact		Duration		Self-control	
		Before nursing	After nursing	Before nursing	After nursing	Before nursing	After nursing
Observation	15	8.07 ± 1.62	3.87 ± 0.92	7.60 ± 1.40	3.20 ± 1.01	4.80 ± 1.32	6.80 ± 1.21
Control	15	7.33 ± 1.80	5.27 ± 0.88	8.27 ± 1.22	4.67 ± 1.05	4.73 ± 1.44	5.00 ± 1.07
*t*		1.172	4.261	1.387	3.898	0.132	4.323
*P*		0.251	＜0.001	0.176	0.001	0.896	＜0.001

Group	*n*	Treatment control		Symptoms		Attention	
		Before nursing	After nursing	Before nursing	After nursing	Before nursing	After nursing
Observation	15	7.20 ± 1.08	7.87 ± 1.41	7.07 ± 1.10	5.93 ± 01.22	7.00 ± 0.76	7.40 ± 0.83
Control	15	6.87 ± 1.13	7.40 ± 1.24	7.27 ± 0.96	5.80 ± 1.01	7.20 ± 1.52	7.20 ± 0.94
*t*		0.827	0.963	0.530	0.325	0.456	0.618
*P*		0.415	0.344	0.600	0.748	0.652	0.542

Group	*n*	Disease awareness		Emotion		Total points	
		Before nursing	After nursing	Before nursing	After nursing	Before nursing	After nursing
Observation	15	4.07 ± 1.49	7.27 ± 0.70	7.33 ± 0.90	3.93 ± 0.59	52.13 ± 8.94	21.60 ± 2.69
Control	15	4.33 ± 0.82	5.93 ± 0.70	7.07 ± 1.22	4.93 ± 0.80	51.47 ± 12.48	26.00 ± 5.03
*t*		0.609	5.189	0.680	3.892	0.168	2.987
*P*		0.547	＜0.001	0.502	0.001	0.868	0.006

**Table 2:** Comparison of nursing cooperation between the two groups of patients (*n* (%)).

Group	*n*	Compliance	Basic compliance	Noncompliance	Overall compliance rate
Observation	15	12 (80.00)	3 (20.00)	0 (0.00)	15 (100.00)
Control	15	4 (26.67)	10 (66.67)	1 (6.67)	14 (93.33)
*χ* ^2^					1.034
*P*					0.309

**Table 3:** Comparison of ESCA scores between the two groups of patients ($\bar{x}$ ± *s*, points).

Group	*n*	Self-concept (0∼36 points)		Self-responsibility (0∼32 points)		Self-care skill (0∼48 points)	
		Before nursing	After nursing	Before nursing	After nursing	Before nursing	After nursing
Observation	15	18.87 ± 3.62	28.47 ± 3.94	20.07 ± 2.99	27.20 ± 4.96	18.53 ± 4.67	37.47 ± 5.83
Control	15	18.47 ± 3.66	23.67 ± 4.22	17.80 ± 5.54	22..00 ± 3.19	19.40 ± 6.12	28.67 ± 5.04
*t*		0.301	3.219	1.394	3.284	0.436	4.242
*P*		0.766	0.003	0.174	0.003	0.666	＜0.001

Group	*n*	Health knowledge level (0∼56 points)		Total score (0∼172 points)			
		Before nursing	After nursing	Before nursing	After nursing		
Observation	15	28.87 ± 3.64	44.87 ± 4.87	96.40 ± 17.56	121.47 ± 10.41		
Control	15	27.73 ± 4.08	38.87 ± 4.22	100.87 ± 13.74	105.40 ± 8.63		
*t*		0.803	3.606	0.776	4.600		
*P*		0.429	0.001	0.444	＜0.001		

The article "Effects of Mind Mapping Combined with Microvideo Explanation on Disease Perception Control and Nursing Cooperation during Membrane Induction Therapy in Patients with Infectious Nonunion after Tibial Trauma" was retracted in 2024. Reasons: signs of a paper mill; suspected computer-generated content; unreliable results or conclusions; lack of ethics approval or compliance.

## Data Availability

The data can be obtained from the corresponding author upon reasonable request.
